The article "Pilot study of fractal dimension analysis of osteogenesis for bone substitute materials of Bio-Oss in lateral sinus augmentation" was published in 2023. Journal: PLoS One.

# Pilot study of fractal dimension analysis of osteogenesis for bone substitute materials of Bio-Oss in lateral sinus augmentation

**DOI:** 10.1371/journal.pone.0296248

**Published:** 2023-12-29

**Authors:** Cai Wen, Qing Zhang

**Affiliations:** 1 Department of Oral Implantology, The Affiliated Stomatology Hospital, Southwest Medical University, Luzhou, Sichuan, China; 2 Department of VIP Dental Service, The Affiliated Stomatology Hospital, Southwest Medical University, Luzhou, Sichuan, China; 3 Luzhou Key Laboratory of Oral & Maxillofacial Reconstruction and Regeneration, The Affiliated Stomatology Hospital, Southwest Medical University, Luzhou, Sichuan, China; 4 Institute of Stomatology, Southwest Medical University, Luzhou, Sichuan, China; 5 Department of Nosocomial Infection Control, The Affiliated Hospital, Southwest Medical University, Luzhou, Sichuan, China; International Medical University, MALAYSIA

## Abstract

**Background:**

Fractal dimension (FD) analysis has been proposed and validated in osseointegration-related research. The aim of this study was to evaluate the feasibility of FD analysis in the osteogenesis detection of bone substitute materials (BSMs) of Bio-Oss in maxillary lateral sinus augmentation.

**Methods:**

Patients who received lateral maxillary sinus augmentation and underwent grafting with BSMs (Bio-Oss) were included in the study. The cross sections of the BSMs under cone-beam computed tomography (CBCT) at mesial, distal, and sagittal directions were obtained immediately after the graft (T0) and 6 months later (T1), and the obtained images were cropped to include only the BSMs. The FD analysis was performed, and the FD value was obtained by the method of box-counting. Paired t-tests and analysis of variance (ANOVA) were used, and p-values <0.05 was considered statistically significant.

**Results:**

Twelve participants with 22 implants, which were inserted simultaneously after sinus augmentation, were included in this study. A total of 22 mesial, 22 distal, and 14 sagittal images were obtained after FD analysis. The mean FD value and standard deviation at T0 was 1.2860 ± 0.0896, while at T1, it was 1.2508±0.1023; thus, significant differences were detected (p = 0.022). However, the increasing or decreasing trend of FD value was not stable, and no significant difference was detected for FD values of mesial, distal, and sagittal images between T0 and T1. ANOVA indicated that no significant difference was detected among the FD values of mesial, distal, and sagittal images at any timepoint. Differences in FD values between the sexes were not significant either.

**Conclusions:**

Since the FD analysis for the osteogenesis detection of BSMs in maxillary sinus augmentation indicated unstable trends of change, its feasibility is not reliable. The initially rough surface, self-degradation, and volume change of the BSMs during osteogenesis may be the reason for the variation in FD values.

## Introduction

Surgical maxillary sinus augmentation was first proposed by Boyne and James [1] in 1980 and was later improved by Summers [2]. After years of development, this procedure is widely used and is now divided into the lateral and transcrestal approaches. Evidence-based clinical practice guidelines recommend that, when the alveolar ridge has sufficient width and the vertical residual bone height is > 4 mm, the transcrestal approach can be utilized [3]. However, for participants with vertical residual bone height < 4 mm or with a slanted sinus floor, the lateral approach is the more predictable procedure [4, 5].

Histological evidence suggests that bone substitute materials (BSMs) have the potential for osteogenesis, osteoconduction, and osteoinduction [6, 7]. Based on general clinical experience, these BSMs can ossify into mature bone structures approximately 6 months after grafting [8]. Currently, the mineralization of BSMs can only be estimated by the brightness variations of the areas under radiographic examination. Previous studies reported that bone density measurements based on Hounsfield units by cone-beam computed tomography (CBCT) were not reliable [9, 10]. However, due to the deep location of BSMs and clinical operability, there has been no direct gold standard or quantifiable method for evaluating the osteogenic properties and trabecular reconstitution of BSMs. Therefore, it is important to find an available, reliable, and simple tool for evaluating the trabecular and mineralization changes in BSMs under noninvasive conditions.

Fractal dimension (FD) analysis [11–13] is a mathematical evaluation method for complex irregular structures using fractal mathematics, which is used to describe the complex structural patterns of bones. FD analysis assumes that the geometric structure and roughness of an object remain constant, regardless of whether the images are enlarged or shrunken. FD values can express geometric features of these images and can be applied to medical analysis, such as determining cell, bone, blood vessel, and nerve distribution as well as bone regeneration.

Bone has a trabecular structure with a potential geometric pattern [14]. Several methods for measuring bone quality by FD analysis on trabecular number have been proposed and validated [15, 16]. Moreover, it is considered that FD analysis may be more reliable than the traditional Hounsfield element analysis or density estimation [17]. However, to our knowledge, there has been no evidence of whether FD analysis of bone formation can be extended to predict osteogenesis of BSMs, which involve the gradual growth of bone trabeculae that eventually replace the BSMs to form mature bone structures [18, 19]. It is possible that the FD value changes in bone substitutes may be similar to those of natural bone formation, which could then be used as a meaningful indicator to measure the maturity of BSMs.

Thus, the aim of this study was to evaluate the effectiveness and feasibility of FD analysis in predicting osteogenesis in BSMs. In this retrospective study, we acquired CBCT data of the participants both at the time of BSM grafting in lateral sinus augmentation and 6 months postoperatively, and compared whether the growth of bone trabeculae in bone substitutes could obtain significant changes during the bone healing period, by using FD analysis via ImageJ software (NIH, Bethesda, MD, USA). The alternative hypothesis was as follows: The FD value of the BSMs at 6 months postoperatively would be significantly different from that at the time of grafting, and the same time, these variations have a stable trend in each CBCT image sections at different treatment timepoints.

## Methods and materials

### Participant selection

This study was approved by the ethics committee of the Affiliated Stomatology Hospital of Southwest Medical University (Ethical Approval Number: 20220118001), and was carried out in accordance with the Declaration of Helsinki. Participants were selected from among patients who underwent lateral sinus augmentation at the Department of Oral Implantology of the Affiliated Stomatology Hospital of Southwest Medical University from January 2017 to August 2022. The surgeries were performed by the same dental implantologist (CW), and the study was conducted from June 2022 to February 2023 and the image samples were collected during that time.

The inclusion criteria were as follows: signed written informed consent, no history of systemic diseases, the residual alveolar height was between 2-4mm,meeting the indications for lateral maxillary sinus elevation, no previous maxillary sinus-related surgery, and no current pathological changes of the paranasal sinus observed on preoperative CBCT evaluation. We excluded patients with contraindications for implantation and lateral sinus augmentation; a history of maxillary sinus surgery regardless of whether it was successful; patients with systemic diseases that affect bone metabolism, such as Paget’s disease, hyperparathyroidism, hypoparathyroidism, osteogenesis imperfecta, anemia, osteomalacia, renal osteodystrophy, hyperthyroidism, cancer with bone metastasis, severe or chronic renal impairment, and/or use of specific drugs or hormones known to have adverse effects on bone metabolism (e.g., corticosteroids, excess thyroid hormones); patients who experienced immediate complications following sinus lift surgery and implant insertion, developed peri-implant infections such as peri-implant mucositis and peri-implantitis, or fail to achieve osseointegration after the healing phase of inserted implants, etc.

### Surgical procedure

Lateral sinus augmentation operation was performed under local anesthesia and strict aseptic conditions. After the flap in the maxillary posterior zone was dissected and elevated, a trapezoidal fenestration was carefully created in the lateral bone wall of the maxillary sinus with a Dentium Advanced Sinus Kit drill (Dentium, Seoul, Korea), and the mucoperiosteal membrane of the maxillary sinus (Schneiderian membrane) was carefully separated using the lifting tool. Care was taken to ensure that there was no obvious rupture of the Schneiderian membrane. BSMs (Bio-oss, Geistlich, Switzerland) was mixed with the participant’s autologous blood and inserted beneath the elevated membrane. The quantity of BSM administered was approximately 0.25cc of Bio-Oss per elevated dental position. After grafting, the implants were inserted simultaneously.

After grafting and implantation, the tissue flap was sutured with a nylon thread under tension-free conditions. All participants were treated with antibiotics for 3‒4 days after the operation, and glucocorticoids were administered for patients with severe swelling reactions.

### Acquisition of region of interest

All patients were examined at a same timeline. CBCT was performed immediately after surgery, and the time-point was set as T0 (immediately after the graft). CBCT images were captured using a KODAK CBCT System (Kodak, NY, USA). Imaging was performed using 90 KV voltage, 10 mA, and 8-s exposure time. CBCT was performed again 6 months after grafting (T1). Dental imaging software (Kodak, NY, USA) for the CBCT equipment was used for radiography analysis on a multi-plane reconstruction window.

To obtain coronal section images of the same region, the cross-section was set at 1 mm mesial and 1 mm distal to every implant and was adjusted along the tangential direction of the dental arch curve and the long-axis direction of the inserted implant. Care was taken to ensure that the body of the implant was not included in the coronal section image (Fig 1). In the screenshot taken at T1, the same positioning policy was used. The image was exported in the format of a TIFF file and named using the participant’s name, tooth position, mesial or distal, and T0 or T1.

**Fig 1:** Acquisition of the mesial and distal direction image. (a) The cross-section was set at 1 mm mesial and 1 mm distal to every implant and was adjusted along the tangential direction of the dental arch curve and the long-axis direction of the inserted implant; (b) Then, a screenshot of the coronal section image of the grafted bone-substitute material was obtained and exported.

We then attempted to obtain an image in the sagittal direction. If more than one implant was placed, the cross-section connected the centers of the two implants. If only one implant was placed, the cross-section direction was perpendicular to the tangent of the dental arch at the point where the implant was located (Fig 2). The same positioning policy was also used repeatedly at T1. The images of the sagittal plane were captured and saved in TIFF format and named using the participant’s name, tooth position, sagittal, and T0 or T1.

**Fig 2:** Acquisition of the sagittal direction image. (a) The cross-section line connects the centers of the two implants; (b) the corresponding sagittal image screenshot was obtained.

We evaluated screenshots taken at T0 and T1 to ensure that they had the same position, angle, and size, and the region of interest (ROI) from the obtained image was intercepted; the cropped ROI image was set to a rectangular shape with height and width between 40 and 100 pixels, respectively. It was necessary to ensure that the participant’s original bone structure and metal structure were not included in the intercepted image, and that only the image of the grafted BSM was selected.

### FD value calculation

The FD analysis of the ROI adopted the geometric counting method of White and Rudolph using ImageJ software (NIH, Bethesda, MD,USA). First, the obtained image was blurred by means of a Gaussian filter, and the brightness change caused by soft tissue was eliminated by the blurring. Then, the original image was subtracted from the blurred image to obtain an image with only trabecular topology. A grey value of 128 was added to each image to obtain an image with an average pixel value of 128. After these transformations, the interference from irrelevant soft structures was removed from the obtained image. The transformation of binarization, erosion, dilatation, inversion, and skeletonization was carried out using ImageJ software, and images with only the pixel center line were obtained (Fig 3).

**Fig 3:** Process of fractal dimension analysis of bone substitute materials grafted in lateral sinus augmentation by ImageJ. (a) acquired images, (b) selection of region of interest in the yellow square, (c) the chosen area, (d) blurred image to remove the influence of soft tissue, (e) image subtraction, (f) increased to 128 Gy level, (g) binarization, (h) erosion, (i) dilation, (j) image color inversion, and (k) image skeletonization.

The FD value calculations were completed using the ImageJ “box-counting function,” as previously described [14, 20]. Squares of 2-, 3-, 4-, 6-, 8-, 12-, 16-, 32- and 64 pixels were placed on the image. The total number of squares containing trabeculae for each pixel of different size was measured. A logarithmic scale diagram of the values was drawn. FD values were calculated by measuring the slope of a line aligned with the plotted points on the graph. The imaging cropping processor could identify individual participants during image collection, but did not participate in the analysis of the data.

### Statistical analysis

The demographic data, information of each image, and the obtained FD value of the participants were recorded in Excel (Microsoft, Redmond, WA, USA) for subsequent statistical analysis using SPSS v23.0 (IBM Corp, Armonk, NY, USA) software. Paired t-tests were used to compare the mesial (FD_M_), distal (FD_D_), sagittal (FD_S_), and overall (FD) values at T0 and T1.

Shapiro‒Wilk and Levene’s tests were conducted to confirm the normal distribution and homogeneity of variance of the data. Analysis of variance (ANOVA) was used to compare the effects between different sites and the sexes on the change in the FD value. Statistical significance was set at P < 0.05.

## Results

Twelve participants with 22 augmented sites by the lateral approach were included in this study. The average age of the participants was 55.1 ± 6.5 years (Table 1). The concrete data of the augmented implant sites were indicated in Table 2.

**Table 1:** Demographic characteristics of participants.

Characteristic	Participants	Implants	Mean Age
Male	8	17	55.6±7.7
Female	4	5	54.0±3.4
Overall	12	22	55.1±6.5

**Table 2:** Data of BSMs augmented tooth position for each participant.

Participants (Sex)	Age	Augmented Tooth Position
1#Female	59	16,17
2#Male	62	15,16
3#Male	56	16,17
4#Female	53	17
5#Male	50	26,27
6#Male	69	26
7#Male	55	16,17,26,27
8#Male	57	15,16, 26,27
9#Male	53	16
10#Male	43	26
11#Female	52	26
12#Female	52	25

At T0 and T1, the mean FD values (±standard deviation) were 1.2674±0.1070 and 1.2281±0.1034, respectively. The FD values of subgroups in the mesial, distal, and sagittal planes are shown in Table 3. FD data from all groups (mesial, distal, sagittal, and overall) showed a normal distribution and homogeneity of variance. The FD values of every site at T0 and T1 were shown in Fig 4.

**Fig 4:** Fractal dimensional values at T0 and T1 for included mesial, distal, and sagittal images. (a) FD values of mesial images, (b) FD values of distal images, and (c) FD values of sagittal images.

**Table 3:** FD values of BSMs in different ROIs and time.

	FD_M_	FD_D_	FD_S_	Overall FD	P_2_
**N.**	22	22	14	58	
**Up N.**	6	7	6	19	
**Down N.**	16	15	8	39	
T_0_	1.2625±0.1022	1.3031±0.0919	1.2192±0.1225	1.2674±0.1070	0.067
T_1_	1.2405±0.0995	1.2716±0.0772	1.1404±0.0973	1.2281±0.1034	0.000*
P_1_	0.416	0.229	0.062	0.022*	

FD: fractal dimension; T_0_: The time point at lateral sinus grafting; T_1_: 6 months after sinus grafting; the footnote of M denote mesial, D denote distal, S denote sagittal; P_1_:FD values comparison between T_0_ and T_1_ at the same ROI (paired t-test); P_2_:FD values comparison between different ROI at the same time (ANOVA)

* denotes significant difference.

Out of 58 BSM-augmented sites, 19 sites showed increased FD values, while 39 sites showed decreased FD values from T0 to T1. The paired t-test showed that there were significant differences between the FD values of the overall participants at T0 and T1 (P = 0.022), while for all other groups (mesial, distal, and sagittal), no significant difference was detected. One-way ANOVA indicated that there was no significant difference in FD values among the mesial, distal, and sagittal images at T0 (P = 0.617); however, a significant difference at T1 (P = 0.000) was observed.

At T0, the FD values of female participants were higher than those of male participants, although the difference was not statistically significant. At T1, on the contrary, the FD value in males was higher than that of women, and the difference was not statistically significant. During the healing period from T0 to T1, FD values decreased in both women and men, and the difference was not statistically significant (Table 4).

**Table 4:** FD values of bone substitute materials of different genders and time.

	FD_Fe_	FD _Ma_	P_2_
**T**_**0**_	1.2709±0.1152	1.2663±0.1056	0.891
**T**_**1**_	1.2154±0.0850	1.2322±0.1092	0.602
**N**	14	44	
**P**_**1**_	0.112	0.089	

FD: fractal dimension; T_0_:Time point at lateral sinus grafting; T_1_:6 months after sinus grafting; the footnote of Fe denote female, Ma denotes male; P_1_: FD values comparison between T_0_ and T_1_ (paired t-test); P_2_: FD values comparison between different genders at the same time (two-sample test).

## Discussion

In this study, we evaluated the feasibility of FD analysis to predict osteogenesis of BSMs. Although there was a significant difference in total FD values between T0 and T1, there was no significant difference in the FD values of mesial, distal, or sagittal images. More importantly, the trend of increasing and decreasing of FD values from T0 to T1 was not uniform. Thus, the statistical difference of overall FD value comparison loses its predictive value.

Lateral maxillary sinus augmentation is currently considered a predictable implant bone-augmentation method [21, 22].The outcomes of lateral wall sinus augmentation is highly predictable as measured by surgical success and implant survival. If appropriate BSMs are selected and the inserted implant can achieve good primary stability, the implant survival rate is expected to exceed 95% [23, 24].Secondly, complications are rare for experienced dentists, and those that occur during and after sinus grafting procedures are mostly local and easily remedied [25].

However, the time needed for mineralization of bone substitutes remains quasi-empirical, and the quality of newly formed bone is unpredictable. The virtual density measurement method using CBCT software is not stably repeatable [26]. In addition, different BSMs [27, 28] (such as hydroxyapatite, tricalcium phosphate, and deproteinized bovine bone) made by different manufacturers usually have varied initial densities. Detumescence of mucosal edema may change the volume of the grafting material, so that density variation cannot be used as a simple indicator of mineralization of the bone substitute. At the same time, artifacts arising from the metal implants interfere with the accuracy of bone density measurement.

FD analysis is a mathematical method for evaluating irregular complex structures. The value derived quantitatively by this method is defined as the FD value [29]. Du Bois Reimond first proposed the concept of continuous non-distinguishable functions in 1875 [30]. The term “fractal” comes from the Latin word “fractus,” meaning “fractured.” To measure the complexity of these structures, it is necessary to count the number of components on a definite scale. It is mathematically expressed by FD = log n / log ε, where n is the number of components and ε is the defined scale [31].

FD analysis differs from traditional geometric analysis methods and can be used to evaluate structures at different scales. Many phenomena in life, such as the shape of leaves, the distribution of blood vessels in the human body, and the growth of bone trabeculae, can be regarded as fractal sets. The FD values are not related to density, only to the complexity of the image. The higher the FD value, the more complex is the disorder of its structure. Fractal analysis has been widely used in computer science. Currently, the applicable fractal analysis software includes Scion Image, Tasplus, NRecon, and ImageJ. ImageJ [32] is a powerful, free, image-processing software, developed by the NIH and based on Java, and is widely used in medical research.

Several methods can be used for FD calculation, such as the power spectral density, triangular prism surface area, blanket method, intensity difference scaling or variogram, and box-counting algorithm. Of the methods applying FD analysis to medical image analysis, the computer program proposed by White & Rudolph is the most frequently used method for bone-related analysis [33, 34]. It measures the morphological features of bone and details the steps of image processing flow standardization to highlight the trabecular structure and eliminate the influence of soft tissue. It uses Gaussian filtering and image fusion and then converts the trabecular structure into a digital image through binarization, corrosion, expansion, and skeletonization. After the image processing process, the topological structure of the bone trabecula is converted into the FD value using a box-counting algorithm.

Currently, the main applications of FD analysis in the field of dentistry are related to the prediction of implant osseointegration [35, 36], peri-implant inflammation [37], periodontitis [38], osteoporosis [39], etc. Southard et al. [12] indicated that FD correlated positively with alveolar bone mineralization; with the increase in bone mineral density, FD also increased, and the average FD decreased in X-ray photographs of decalcified human alveolar bone. Wilding et al. [40] measured the FD value of a panoramic image of an implant-fixed denture and analyzed the bone structure mesial and distal to the implants; the FD value at the implant neck area increased significantly with remodeling of the bone trabecular 2 years after implantation. Lee et al. [41] studied the relationship between the FD value of peri-implant bones and primary stability of implants using resonance frequency analysis. They found a significant correlation between the FD values and implant stability and stated that the FD value may be an effective predictor of the initial implant stability. Although fractal analysis has been used to evaluate osseointegration between implants and bones, few studies have evaluated the trabecular structure formation of BSMs.

The mineralized and osteogenesis process of BSM may differ from that of natural bone. These materials have the effect of osseoconduction and act as a scaffold, into which blood vessels and cells of the host enter. Specifically, osteoblasts infiltrate and deposit new bone, and bone cells differentiated from mesenchymal progenitor cells gradually replace the BSM [42, 43]. During this process, the formation of trabecular bone structures may lag behind the rate of the bone’s preliminary maturation. Although under normal circumstances, after a healing phase of approximately 6 months, the BSM is considered to have reached the maturity of natural bone, and there are still no reliable noninvasive tests to confirm bone remodeling in individuals. The results of the present study rejected the null hypothesis: the variations in the FD value of the BSMs 6 months postoperatively did not have a stable trend. The feasibility of FD analysis of osteogenic detection of BSMs thus remains unclear.

It has been assumed that the higher the box-counting value, the more complex the trabecular bone, and that a decrease in bone mineral density corresponds to the decrease in FD, as verified by previous studies [15, 37, 41, 44, 45]. However, in the present study, the mean FD values actually decreased after 6 months of osteogenesis, indicating that the methods used in previous studies are not appropriate for BSMs. The differences in the findings of our own and these previous studies may be due to differences between two-dimensional (2D) and three-dimensional (3D) images, and differences in mineralization processes between BSMs and natural bone:

1. In this study, we used 3D CBCT images, which differ from the 2D images, such as panoramic films and periapical images, used in most previous studies. The formation of bone trabeculae occurs in 3D space, and 2D images obtained from 3D data may eliminate some information on spatial distribution of bone trabeculae. Although CBCT is considered to be more accurate than panoramic imaging in evaluating bone quality (due to its 3D and high-resolution images, with low radiation dose and low distortion), it may cause partial loss of spatial data when describing bone trabecular structure as compared with 2D images. This issue requires further clarification and confirmation.
2. When we used FD analysis in this study, we calculated the FD value of the topological structure formed by the mixture of the initial BSMs, the gradually degraded BSMs, and the newly formed bone trabeculae. The increased complexity of the new bone trabecular structure may be less than the decreased complexity caused by the degradation of BSM. Therefore, we consider that White and Rudolph’s method of FD analysis may not be entirely suitable for BSMs, or that the mechanism of BSM osteogenesis may differ from that of natural bone; thus, changes in the structural profile of BSMs and the generation of trabecular bone structures may make FD analysis ineffective.

### Limitation

With the advancement of bioengineering, numerous novel BSMs exhibiting excellent osteogenic properties have emerged [46, 47]. However, in this study, we selected only one type of bone substitute material (BSM) of Bio-Oss due to material availability, experimental design and other related reasons. Based on the principle of minimal radiation, although most BSMs did not achieve complete bone transformation after six months of implant bone healing phase [48, 49], patients were scheduled for radiographic examination at two time points: immediately after surgery and six months later. This was due to their refusal for longer follow-up and repeated exposure to radiation detection. As the aim of this study was to validate the use of FD analysis in assessing the osteogenic result of BSM, the degree of bone integration did not compromise the result of our findings.

## Conclusion

FD analysis were unable to demonstrate the effectiveness of FD analysis in the osteogenesis detection of bone mineralization and the growth of bone trabeculae of BSMs after maxillary lateral sinus augmentation. The irregular increasing or decreasing variations of FD values of BSMs may be related to its mineralization and self-degradation during the osteogenesis process.

## Supporting information

S1 File The raw fractal dimension analysis data of this research. (XLS)

## Abbreviations

FD: fractal dimension
BSM: bone substitute materials
CBCT: cone-beam computed tomography
